# SMAD-PI3K-Akt-mTOR Pathway Mediates BMP-7 Polarization of Monocytes into M2 Macrophages

**DOI:** 10.1371/journal.pone.0084009

**Published:** 2013-12-20

**Authors:** Crystal Rocher, Dinender K. Singla

**Affiliations:** Biomolecular Science Center, Burnett School of Biomedical Sciences, College of Medicine, University of Central Florida, Orlando, Florida, United States of America; University of Texas Medical Branch, United States of America

## Abstract

Previously we demonstrated that bone morphogenetic protein-7 (BMP-7) treatment polarizes monocytes into M2 macrophages and increases the expression of anti-inflammatory cytokines. Despite these findings, the mechanisms for the observed BMP-7 induced monocyte polarization into M2 macrophages are completely unknown. In this study, we demonstrate the mechanisms involved in the polarization of monocytes into M2 macrophages. Apoptotic conditioned media (ACM) was generated to mimic the stressed conditions, inducing monocyte polarization. Monocytes were treated with ACM along with BMP-7 and/or its inhibitor, follistatin, for 48 hours. Furthermore, an inhibitor of the PI3K pathway, LY-294002, was also studied. Our data show that BMP-7 induces polarization of monocytes into M2 macrophages while significantly increasing the expression of anti-inflammatory markers, arginase-1 and IL-10, and significantly (p<0.05) decreasing the expression of pro-inflammatory markers iNOS, IL-6, TNF-α and MCP-1; (p<0.05). Moreover, addition of the PI3K inhibitor, LY-294002, significantly (p<0.05) decreases upregulation of IL-10 and arginase-1, suggesting involvement of the PI3K pathway in M2 macrophage polarization. Next, following BMP-7 treatment, a significant (p<0.05) increase in p-SMAD1/5/8 and p-PI3K expression resulting in downstream activation of p-Akt and p-mTOR was observed. Furthermore, expression of p-PTEN, an inhibitor of the PI3K pathway, was significantly (p<0.05) increased in the ACM group. However, BMP-7 treatment inhibited its expression, suggesting involvement of the PI3K-Akt-mTOR pathway. In conclusion, we demonstrate that BMP-7 polarizes monocytes into M2 macrophages and enhances anti-inflammatory cytokine expression which is mediated by the activated SMAD-PI3K-Akt-mTOR pathway.

## Introduction

Atherosclerosis, an inflammatory disease that results in hardening and narrowing of large and small arteries due to plaque formation, is the leading cause of myocardial infarction and stroke and affects millions of people every year [1]–[4]. Previous data suggest that the inflammatory response that occurs during atherosclerosis development can determine the severity of the disease and its progression [4]. During inflammation, monocytes migrate to the injured area and differentiate into macrophages [1], [2]. Within a pathological environment, the role of macrophages is multi-faceted and complex and plays a central role to the physiology of the disease.

There are two main categories of macrophages known as classical M1 macrophages and alternative M2 macrophages [1], [5]. Classical M1 macrophages are pro-inflammatory and secrete such factors as iNOS, IL-6, TNF-α, and MCP-1, which can enhance the inflammatory response and result in disease progression. Conversely, alternative M2 macrophages are anti-inflammatory and secrete factors such as IL-10 and arginase-1 [5]–[7]. Specifically, published data have suggested M2 macrophages promote tissue repair and wound healing [1], [5]. To this end, identification of mechanisms used to direct the ratio of M1 and M2 macrophages toward a greater percentage of M2 macrophages following monocyte polarization may offer novel, potential treatment options for patients suffering from inflammatory diseases such as atherosclerosis.

Bone morphogenetic protein-7 (BMP-7), a signaling molecule belonging to the transforming growth factor beta (TGF-β) superfamily, works through activation of BMPR2, which results in phosphorylation of R-SMAD1/5/8 and activation of downstream mediators in the SMAD pathway. Evidence provided suggest this occurs in chondrocytes, mesenchymal stem cells and kidney cells as well as disease models such as osteoarthritis, diabetic nephropathy and renal injury [8]–[10]. However, the mechanisms of BMP-7-induced monocyte polarization into M2 macrophages remain unknown. Therefore, we hypothesized that following BMP-7 treatment, M2 macrophage polarization occurs due to the activation of the PI3K-Akt-mTOR pathway. In the present study, our data demonstrate that following treatment with BMP-7, expression of p-SMAD1/5/8 significantly increased resulting in increased expression and activation of p-PI3K. Furthermore, we identified that activation of PI3K lead to downstream activation of p-Akt and p-mTOR, following the initiation of the PI3K-Akt-mTOR pathway. Follistatin, a BMP-7 inhibitor, significantly reduced M2 macrophage polarization as well as PI3K-Akt-mTOR pathway suggesting its role in polarization. Additionally, LY-294002, an inhibitor of the PI3K pathway, was studied and corroborated the effects of BMP-7 on M2 macrophage polarization through the examination of M2 macrophage released anti-inflammatory cytokines, IL-10 and arginase-1.

## Materials and Methods

### In-vitro cell culture model

As per manufacturer's instructions, human monocytes (THP-1 cells) purchased from ATCC, were grown in 25 cm^2^ flasks and cultured every other day in RPMI 1640 (ATCC) supplemented with 10% fetal bovine serum and 0.05 mM β-mercaptoethanol [5].

### Stress induced injury model

Apoptotic conditioned media (ACM) was generated and cell concentration used for monocytes was previously reported by us [5], [11]. In brief, 60 mm tissue culture dishes were each plated with 5×10^5^ H9c2 cardiomyoblasts for 24 hours. The cells were then treated with 400 uM H_2_O_2_ for 2 hours. Following treatment, media was collected, filtered, labeled ACM, and stored for future use.

### Monocyte polarization treatment

Monocytes were divided into the following groups: Control (monocytes cultured in normal media), ACM (monocytes cultured in normal media + ACM (40% v/v)), ACM+BMP7 (monocytes cultured in normal media + ACM (40% v/v) +660 ng/ml BMP-7), and ACM+BMP7+Follistatin (Foll) (monocytes cultured in normal media + ACM (40% v/v) + 660 ng/ml BMP-7+500 ng/ml Foll). Experimental conditions and mouse BMP-7 (Bioclone, San Diego, CA) and follistatin (Sino Biological, Beijing, China) concentrations were used as previously reported by us [5]. Briefly, monocytes were initially plated in a 24 well plate with 40,000 cells per well for 24 hours for stabilization. The cells were then treated based on the aforementioned groups for an additional 48 hours.

### LY-294002 treatment

The PI3K inhibitor, LY-294002, was used as previously reported [12]. The monocytes were divided into the following groups: Control (monocytes cultured in normal media), ACM (monocytes cultured in normal media + ACM (40% v/v)), ACM+BMP7 (monocytes cultured in normal media + ACM (40% v/v) + 660 ng/ml BMP-7), and ACM+BMP7+LY) (monocytes cultured in normal media + ACM (40% v/v) +660 ng/ml BMP−7+40 µM LY). As stated above, the monocytes were plated in a 24 well plate with 40,000 cells per well for 24 hours. Then, the cells were treated according to the above groups for 48 hours and next used for experimental analysis.

### Immunohistochemistry of BMPR2 and macrophage markers

As previously reported, cells were removed from the 24 well plate, centrifuged and used to make smears on ColorFrost Plus glass slides [5]. The smears were fixed with 4% paraformaldehyde and blocked with either 10% normal goat serum or normal donkey serum (Vector Labs) for one hour at room temperature. Following blocking, the smears were incubated with primary antibodies for either anti-CD14, anti-iNOS, anti-CD206, anti-arginase-1, or anti-BMPR2 overnight at 4°C. Next, appropriate secondary antibodies, goat anti-rabbit Alexa 568 or donkey anti-goat Alexa 488, were added for 1 hour at room temperature. Finally, the smears were stained with DAPI (4′, 6-diamidino-2-phenylindole) (Vector Labs) and cover-slipped. The slides were analyzed under an Olympus fluorescent microscope.

### Pro and anti-inflammatory cytokine ELISAs

ELISA kits were purchased from Raybiotech and used to quantify anti-inflammatory (IL-10) and pro-inflammatory (IL-6, TNF-α, and MCP-1) cytokine expression. Following treatment, the culture media was isolated from each group, centrifuged, and the supernatant collected. The supernatant was then added to pre-coated strips and the ELISAs were performed as per manufacturer's instructions and as previously reported [5].

### Western blot analysis

Western blot was performed as previously reported [12]. In brief, cells were collected, centrifuged, and lysed on ice for 30 minutes in RIPA buffer supplemented with protease inhibitor cocktail, PMSF, sodium orthovanadate and sodium fluoride. Protein concentration was estimated for each cell lysate using the Bio-Rad protein assay and read on a microplate reader at 595 nm. Following protein concentration determination, 100 µg of the prepared protein samples were loaded and run on an 8 or 10% sodium-dodecyl sulfate polyacrylamide gel at 150 V for 60 to 80 minutes depending on the molecular weight of the proteins to be separated. Next, proteins were transferred onto a PVDF membrane (Bio-Rad) which was then blocked with 5% milk and incubated with the primary antibodies p-SMAD1/5/8 (Cell Signaling, 1∶1000), p-PI3K (Cell Signaling, 1∶1000), Total PI3K (Cell Signaling, 1∶1000), p-Akt (Cell Signaling, 1∶1000), p-PTEN (Cell Signaling, 1∶1000), p-mTOR (Cell Signaling, 1∶1000) or Total mTOR (Cell Signaling, 1∶1000). Following primary antibody incubation, membranes were washed, incubated with secondary antibody anti-rabbit IgG (Cell Signaling, 1∶1000), and then exposed with a Visualizer. Densitometry analysis was completed with the help of Image J software which allows for the quantification of band intensity. Developed films were scanned and opened using Image J software. A rectangle was placed on each band and the band intensity was analyzed as well as the background intensity. Quantification was determined by subtracting band intensity with background intensity. Protein expression was corrected with a loading control such as β-actin, total mTOR or total PI3K and this by dividing the protein densitometry value by its control. All western blot data is presented as: Protein densitometry/control protein densitometry.

### Statistical analysis

Data was analyzed using One-way analysis of variance (ANOVA) followed by the Tukey Test. Data is presented as a mean ± SEM and statistical significance assigned when p-value <0.05.

## Results

### Expression of BMPR2 increases following treatment with BMP-7 on monocytes

Representative photomicrographs shown in Figure 1A demonstrate BMP-7 receptors (BMPR2) in green (a, f, k, p), CD14 positive monocytes in red (b, g, l, q), total nuclei stained blue (c, h, m, r), merged images of cells positive for BMPR2, CD14 and DAPI (d, i, n, s) and enlarged merged images (e, j, o, t). Quantitative analysis reveals that following treatment with BMP-7, monocytic BMPR2 expression is significantly enhanced compared to the control and ACM groups (Figure 1B). Additionally, BMPR2 expression was significantly inhibited in the ACM+BMP7+Foll group compared to the ACM+BMP7 groups suggesting follistatin blocks BMPR2 upregulation through inhibition of normal BMP-7 mediation.

**Figure 1:** Treatment with BMP-7 increases expression of BMPR2 on monocytes. Left panel **A** shows representative photomicrographs of anti-BMPR2 in green (a, f, k, p), anti-CD14 in red (b, g, l, q), DAPI in blue (c, h, m, r), merged images (d, i, n, s) and enlarged merged images (e, j, o, t). Scale bar  = 50 µm. Right histogram **B** shows quantitative analysis of CD14 positive cells expressing BMPR2 with a significant increase in the ACM+BMP7 group compared to Control, ACM and ACM+BMP7+Foll groups. *p<0.05 vs Control, #p<0.05 vs ACM, $p<0.05 vs ACM+BMP7, n = 6.

### Expression of BMPR2 increases following treatment with BMP-7 on M2 macrophages

Figure 2A is representative images of cells positive for BMPR2 in green (a, f, k, p), CD206 (an M2 macrophage marker) in red (b, g, l, q), total nuclei in blue (c, h, m, r), merged images (d, i, n, s) and enlarged merged images (e, j, o, t). BMPR2 expression was significantly enhanced on polarized M2 macrophages in the ACM+BMP7 groups relative to control and ACM groups (Figure 2B). However, a significant reduction in BMPR2 expression on M2 macrophages was observed in the ACM+BMP7+Foll group compared with the ACM+BMP7 group (figure 2B).

**Figure 2:** Expression of BMPR2 is increased in M2 macrophages following treatment with BMP-7. Left panel **A** shows representative photomicrographs of anti-BMPR2 in green (a, f, k, p), anti-CD206 in red (b, g, l, q), DAPI in blue (c, h, m, r), merged images (d, i, n, s), and enlarged merged images (e, j, o, t). Scale bar  = 50 µm. Right histogram **B** shows quantitative analysis of CD206 positive cells expressing BMPR2 with a significant increase in the ACM+BMP7 group compared to Control, ACM and ACM+BMP7+Foll groups. *p<0.05 vs Control, #p<0.05 vs ACM, $p<0.05 vs ACM+BMP7, n = 5–6.

### Treatment with BMP-7 decreases expression of pro-inflammatory markers

Representative photomicrographs shown in Figure 3A demonstrate iNOS positive M1 macrophages in red (a, e, i, m), total nuclei in blue (b, f, j, n), merged images in pink (c, g, k, o), and enlarged merged images (d, h, l, p) for all control and experimental groups. iNOS positive M1 macrophage concentrations were significantly enhanced in the ACM and ACM+BMP7+Foll groups compared to control (Figure 3B). However, the number of M1 macrophages was significantly decreased in the BMP-7 treated group relative to the ACM treated group (Figure 3B). Additionally, compared with the ACM+BMP7 treatment group, M1 macrophages were significantly enhanced in the ACM+BMP7+Foll group (Figure 3B) suggesting BMP-7 prevents monocyte to M1 macrophage polarization.

**Figure 3:** Treatment with BMP-7 decreases expression of M1 macrophage marker, iNOS, as well as pro-inflammatory cytokines. Left panel **A** shows representative photomicrographs of anti-iNOS in red (a, e, i, m), DAPI in blue (b, f, j, n), merged images (c, g, k, o) and enlarged merged images (d, h, l, p). Scale bar  = 50 µm. Histogram **B** shows quantitative analysis of the percentage of cells expressing iNOS with a significant decrease in the control and ACM+BMP7 and groups and a significant increase in the ACM and ACM+BMP7+Foll groups; n = 5–6. Histogram **C** shows quantitative analysis of expression of IL-6 with a significant decrease in the ACM+BMP7 group; n = 5–6. Histogram **D** shows quantitative analysis of expression of TNF-α with also a significant decrease in the ACM+BMP7 group; n = 4–6. Histogram **E** shows quantitative analysis of MCP-1 with also a significant decrease in the ACM+BMP7 group; n = 5–7. *p<0.05 vs Control, #p<0.05 vs ACM, $p<0.05 vs ACM+BMP7.

Quantitative analysis of pro-inflammatory cytokine data including IL-6, TNF-α and MCP-1 is represented in Figures 3C, D and E, respectively. Data suggest a significant increase in IL-6, TNF-α and MCP-1 expression in the ACM group compared with control (Figure 3C, D, and E). However, this increased concentration of pro-inflammatory cytokines was significantly abolished following BMP-7 treatment (Figure 3C, D, and E). Moreover, follistatin treatment resulted in significantly increased expression of IL-6, TNF-α and MCP-1 (Figure 3C, D, and E).

### Anti-inflammatory expression increases following treatment with BMP-7

Representative photomicrographs demonstrating CD206 positive M2 macrophages in red (a, e, i, m), total nuclei stained blue (b, f, j, n), merged images in pink (c, g, k, o), and enlarged merged images (d, h, l, p) are depicted in Figure 4A. Corresponding quantitative analysis of the percentage of cells positive for the M2 macrophage marker, CD206, reveal a significant increase in the number of M2 macrophages in the ACM+BMP7 group compared to control and ACM groups (Figure 4B). However, the number of M2 macrophages was significantly decreased in the ACM+BMP7+Foll group relative to the ACM+BMP7 group (Figure 4B).

**Figure 4:** Following treatment with BMP-7 polarization of monocytes into M2 macrophages increases as well as expression of anti-inflammatory markers. Left panel A shows representative photomicrographs of anti-CD206 in red (a, e, i, m), DAPI in blue (b, f, j, n), merged images (c, g, k, o) and enlarged merged images (d, h, l, p). Scale bar  = 50 µm. Histogram B shows quantitative analysis of the percentage of cells expressing CD206 with a significant increase in the ACM+BMP7 group and a significant decrease in the ACM and ACM+BMP7+Foll groups; n = 5–6. Histogram C shows quantitative analysis of the percentage of cells expressing Arginase-1 with a significant increase in the ACM+BMP7 group; n = 5–6. Histogram D shows quantitative analysis of the expression of anti-inflammatory cytokine, IL-10, with a significant increase in the ACM+BMP7 group; n = 5–6. *p<0.05 vs Control, #p<0.05 vs ACM, $p<0.05 vs ACM+BMP7.

Anti-inflammatory signaling molecules including arginase-1 and IL-10 were also assessed. Following treatment with BMP-7, a significant increase in the percentage of cells positive for arginase-1 was observed (Figure 4C). However, following follistatin treatment, a significant decreased was detected in the percentage of arginase-1 positive cells compared to the ACM+BMP7 group (Figure 4C). Additionally, levels of IL-10 were significantly increased in the ACM+BMP7 group compared to the control and ACM groups (Figure 4D). Conversely, treatment with follistatin abrogated the increased IL-10 expression following BMP-7 treatment (Figure 4D). Collectively, our data suggest BMP-7 promotes M2 macrophage polarization and anti-inflammatory expression.

### Treatment with LY-294002 inhibits the BMP-7 induced increase in IL-10 and arginase-1

In order to further confirm the role of BMP-7 on M2 macrophage anti-inflammatory cytokine expression through activation of the PI3K pathway, an inhibitor of the PI3K pathway, was used. Figure 5A shows quantitative expression of anti-inflammatory cytokine, IL-10. Following treatment, levels of IL-10 remained the same between the Control and ACM groups; however, they were significantly increased in the ACM+BMP7 group compared to the control and ACM groups (Figure 5A). When treated with LY the increased IL-10 expression significantly decreased compared to the ACM+BMP7 group (Figure 5A). Furthermore, the percentage of arginase-1 positive cells was also examined. Figure 5B shows that there is no significant increase in percentage of positive cells in the Control and ACM group, but when treated with BMP-7, the percentage significantly increased. However, following LY treatment, the percentage of arginase-1 positive cells significantly decreased compared to the ACM+BMP7 group (Figure 5B). This data suggests that treatment with a PI3K inhibitor such as LY decreases expression of anti-inflammatory cytokines which are released by M2 macrophages. Therefore, we interpret that a decrease in these anti-inflammatory cytokines will also affect M2 macrophage polarization, which maybe mediated by the PI3K pathway.

**Figure 5:** Treatment with LY-294002 decreases expression of anti-inflammatory cytokines. Histogram **A** shows quantitative analysis of the expression of anti-inflammatory cytokine, IL-10, with a significant increase in the ACM+BMP7 group; n = 5–6. Histogram **B** shows quantitative analysis of the percentage of cells expressing Arginase-1 with a significant increase in the ACM+BMP7 group; n = 5. *p<0.05 vs Control, #p<0.05 vs ACM, $p<0.05 vs ACM+BMP7.

### BMP-7 promotes activation of SMAD1/5/8 and PI3K

To elucidate mechanisms by which BMP-7 promotes M2 macrophage polarization, mediators of BMP signaling were investigated. Figure 6A, top panel, depicts representative activated Smad1/5/8, downstream effectors of BMP signaling, and corresponding control β-actin blots. Quantitative analysis suggests a significant decrease in activated Smad1/5/8 expression in the ACM group (Figure 6A). Following BMP-7 treatment, phosphorylated Smad1/5/8 (p-Smad1/5/8) expression dramatically increased which was abolished following treatment with follistatin (Figure 6A).

**Figure 6:** Binding of BMP-7 to BMPR2 phosphorylates R-SMAD1/5/8 which activates PI3K. Representative western blot bands (**A**) are shown of p-SMAD1/5/8 and β-actin with densitometric analysis of P-SMAD1/5/8 showing a significant increase of expression in the ACM+BMP7 group and a significant decrease of expression in the ACM and ACM+BMP7+Foll groups. Representative western blot bands (**B**) are shown of p-PI3k and total PI3K with densitometric analysis of p-PI3K showing a significant increase of expression in the ACM+BMP7 group and a significant decrease of expression in the ACM and ACM+BMP7+Foll groups. *p<0.05 vs Control, #p<0.05 vs ACM, $p<0.05 vs ACM+BMP7, n = 5-7.

Representative blots of phosphorylated phosphoinositide 3-kinase (p-PI3K), a enzymatic signaling molecule responsible for promoting cell proliferation, differentiation, and survival, and total PI3K are shown in the top panels of Figure 6B. Activated PI3K expression was significantly decreased in the ACM group compared to control whereas p-PI3K expression was significantly increased following BMP-7 treatment (Figure 6B). However, activated PI3K was significantly decreased in the ACM+BMP7+Foll group compared to the ACM+BMP7 group (Figure 6B).

### Downstream activation of Akt and mTOR occur following BMP-7 treatment

Downstream mediators of the PI3K pathway were investigated to discern mechanisms of PI3K pathway augmentation via BMP-7. Figure 7A-C, top panels, show representative blots of phosphorylated Akt (p-Akt), phosphatase and tensin homolog (p-PTEN), and mammalian target of rapamycin (p-mTOR), respectively. Activated Akt was significantly enhanced in the ACM+BMP7 group whereas a significant decrease in p-Akt expression was noted in the ACM+BMP7+Foll group (Figure 7A). PTEN, an inhibitor of PI3K and subsequent Akt activation, was significantly upregulated in the ACM ad ACM+BMP7+Foll groups compared to the control group (Figure 7B). However, treatment with BMP7 inhibited PTEN activation significantly (Figure 7B). Finally, densitometric analysis of p-mTOR over total mTOR expression revealed a significant increase in expression in the ACM+BMP7 group compared to ACM which was abolished following follistatin treatment (Figure 7C).

**Figure 7:** Activation of PI3K results in phosphorylation of Akt and mTOR and inhibition of the pathway occurs via PTEN. Representative western blot bands (**A**) are shown of p-Akt and β-actin as well as densitometric analysis with a significant increase of expression in the ACM+BMP7 group and a significant decrease of expression in the ACM+BMP7+Foll group. Next, representative western blot bands (**B**) are shown of p-PTEN and β-actin with densitometric analysis showing significant decrease of expression in the ACM+BMP7 group and a significant increase of expression in the ACM and ACM+BMP7+Foll groups. Lastly, representative western blot bands (**C**) are shown of p-mTOR and total mTOR with densitometric analysis showing a significant increase of expression in the ACM+BMP7 group and a significant decrease of expression in the ACM+BMP7+Foll groups. *p<0.05 vs Control, #p<0.05 vs ACM, $p<0.05 vs ACM+BMP7, n = 5–7.

## Discussion

Atherosclerosis, an inflammatory disease leading to arterial wall thickening consequent to plaque formation and accumulation, is the leading cause of myocardial infarction and stroke [4]. Monocytes play an elemental role in the development and progression of inflammatory diseases in that they migrate to damaged areas, divide and differentiate into macrophages. Monocyte differentiation has the potential to yield pro-inflammatory M1 macrophages or anti-inflammatory M2 macrophages. Data provided has suggested the ratio of M1 to M2 macrophages following monocyte polarization can determine the severity and progression of inflammatory disorders [1], [2], [13]. Deciphering the role and mechanisms of monocyte polarization during inflammation has recently gained the attention of the research community. Identification of novel growth factors/molecules used to direct monocyte differentiation and pathways by which this occurs may provide novel therapeutic options for patients with inflammatory diseases such as atherosclerosis.

Bone morphogenic proteins (BMPs) are growth factors, which constitute the largest subset of molecules belonging to the TGF-β superfamily. Signal transduction mechanisms promoted by BMPs occur through activation and oligomerization of BMP receptors (BMPRs) inducing phosphorylation of Smad 1/5/8 and Smad-independent signaling cascades resulting in transcriptional regulation of target genes. Moreover, there are different isoforms of BMPs and the role played by these different BMPs varies from apoptosis, to proliferation, to differentiation [14]. For example, BMP-2 has been shown to induce cardiomyocyte differentiation [14]. Therefore, this is a wide area of research that needs to be further explored in order to determine the effects of different BMPs on Smad and/or PI3K pathway activation and subsequent M2 macrophage polarization. Recently reported, BMP-7 was identified as a novel mediator of monocyte polarization into M2 macrophages [5]. However, the signaling pathway by which BMP-7 promotes M2 macrophage polarization remains obscure. To this end, the current study was undertaken to identify mediators of BMP-7 induced monocyte differentiation and propose a mechanism by which M2 macrophage polarization occurs.

The BMPR2 receptor is directly involved in the BMP-7 ligand induced oligomerization and subsequent signal transduction activity. Under normal and stressed conditions induced by ACM, BMPR2 expression remained unchanged on monocytes and M2 macrophages as evidenced by co-localization of BMPR2/CD14 and BMPR2/CD206, respectively. However, exogenous BMP-7 application resulted in a significant increase in BMPR2 expression on monocytes and M2 macrophages suggesting an increase in BMP-7 signal transduction activity. Several studies have supplied supporting evidence to the current findings indicating an upregulation of BMPR2 expression at 2 days following BMP-7 administration in various models including TNBS-induced colitis [5], [15]. Of note, following treatment with follistatin, an inhibitor of BMP-7 signal transduction, significant upregulation of BMPR2 on monocytes and M2 macrophages was abolished suggesting a direct relation between BMP-7 signaling and upregulation of BMPR2.

A determinant of pathology progression is dependent on macrophage type yields during monocyte differentiation [1], [2], [4], [13], [16]. To this end, M1 macrophage polarization was investigated as well as concentrations of pro-inflammatory cytokines. Treatment with ACM and ACM plus follistatin induced monocyte polarization towards the M1 phenotype, whereas treatment with BMP-7 dramatically decreased M1 macrophage yields suggesting the potential of BMP-7 to prevent monocyte to M1 macrophage polarization. Congruent with increased M1 macrophage concentrations, pro-inflammatory cytokines, IL-6, TNF-α and MCP-1 were significantly increased in the ACM and follistatin groups. Conversely, following BMP-7 administration, concentrations of IL-6, TNF-α and MCP-1 were significantly reduced suggesting a correlation between BMP-7, diminished M1 macrophage polarization, and reduced pro-inflammatory cytokine expression.

Equally important, quantification of anti-inflammatory M2 macrophage polarization revealed a significant higher yield of M2 macrophages following BMP-7 treatment and this increase was adversely augmented following treatment with follistatin. Furthermore, in agreement with M2 macrophage yields, anti-inflammatory markers, arginase-1 and IL-10 were significantly increased following treatment with BMP-7. Data presented suggest, in the presence of BMP-7, monocytes are more readily polarizing into M2 macrophages and expressing anti-inflammatory cytokines but inhibition of BMP-7 by its inhibitor, follistatin, prevents that polarization as well as the enhanced expression of anti-inflammatory cytokines. Our data is in accordance with previous reports demonstrating that, under pathological stressed conditions, monocytes, which exhibit high plasticity, will undergo polarization into macrophages and treatment with certain factors can direct polarization and increase the ratio of M2 macrophages over M1 macrophages [1], [4], [5], [17], [18]. By increasing polarization of M2 macrophages from monocytes and thereby increasing expression of anti-inflammatory markers, the beneficial potential of BMP-7 may include decreasing the progression of the inflammatory response and preventing further injury.

BMP-7 is known to activate the SMAD1/5/8 pathway following binding to BMPR2 but studies have shown that it is also responsible for activation of other non-SMAD pathways such as the PI3K-Akt-mTOR pathway [3], [8], [19]. For example, in granulosa cells, BMP-7 was observed to activate the PI3K pathway resulting in cell survival [3]. Moreover, activation of the PI3K pathway through BMP-7 was also shown in THP-1 cells resulting in increased chemotaxis [19]. Although a correlation between the SMAD1/5/8 and PI3K pathway has been suggested, the importance of these pathways with regards to M2 macrophage polarization following monocyte treatment with BMP-7, has never been reported.

In the present study, our data suggest that BMP-7 upregulates and binds BMPR2, phosphorylates SMAD1/5/8, and activates PI3K, which results in downstream activation of Akt and mTOR as shown in Figure 8. Additional evidence provided demonstrates expression of p-PTEN, an inhibitor of the PI3K pathway, was significantly upregulated in the ACM and ACM+BMP7+Foll groups but was significantly downregulated following BMP-7 treatment suggesting the ability of BMP-7 to not only promote PI3K signaling through upregulated mediators but also by directly blocking inhibition of the signaling cascade [20]. Furthermore, the inhibitor of BMP-7, follistatin, successfully prevented increased p-SMAD1/5/8 expression and significantly decreased expression of PI3K, which is in accordance with previous reports on the role of follistatin as an inhibitor to BMP-7 [21], [22]. Such evidence supports and suggests the necessity of BMP-7 to bind BMPR2 thus activating SMAD1/5/8 and subsequently PI3K.

**Figure 8:** Diagram of the mechanism of BMP-7 monocyte polarization.

Activation of the PI3K pathway controls production of transcriptional factors which regulate key inflammatory cytokines resulting in increased expression of anti-inflammatory markers such as arginase-1 and IL-10 and inhibition of the production of pro-inflammatory markers [20], [23]–[25]. Specifically, in bone marrow derived macrophages, activation of the PI3K pathway resulted in increased polarization of M2 macrophages [26]. Studies have also shown that inhibition of either PI3K or mTOR result in M1 macrophage polarization demonstrating the importance of this pathway in the polarization of monocytes [23], [26]. We suggest that activation of the signaling pathway portrayed in Figure 8 following BMP-7 administration resulted in increased expression of anti-inflammatory cytokines and inhibited expression of pro-inflammatory cytokines, which promoted paracrine effects on monocytes and macrophages yielding increased M2 macrophage polarization.

Moreover, an inhibitor for the PI3K pathway was also examined in the present study to confirm the role of this pathway on M2 macrophage polarization and the release of anti-inflammatory cytokines. BMP-7 treatment significantly increased expression of IL-10 and percentage of arginase-1 positive cells. Interestingly, treatment with LY significantly decreased these levels, suggesting that BMP-7 induced M2 macrophage polarization and the release of anti-inflammatory cytokines are mediated by the PI3K pathway.

Within the present study, we are the first to show, as to the best of our knowledge, the effects of BMP-7 on monocyte polarization and the contributing mechanisms. Collectively, data presented has shown that BMP-7 plays a role in monocyte polarization and can induce M2 macrophage polarization as well as increase expression of anti-inflammatory cytokines. Furthermore, we suggest that mechanisms promoting monocyte polarization following BMP-7 treatment involve activation of the PI3K-Akt-mTOR pathway. In this study, we focused on the effects of BMP-7 on monocyte polarization following 48 hours of treatment, however, further studies will need to be performed involving other time points to fully understand the effects of BMP-7 on PI3K signaling and monocyte polarization.
